The article "Effect of Model Parameters on the Biomechanical Behavior of the Finite Element Cervical Spine Model" was retracted in 2023. Reasons: signs of a paper mill; compromised peer review; unreliable results or conclusions.

# Effect of Model Parameters on the Biomechanical Behavior of the Finite Element Cervical Spine Model

**DOI:** 10.1155/2021/5593037

**Published:** 2021-06-27

**Authors:** Suzan Cansel Dogru, Yunus Ziya Arslan

**Affiliations:** ^1^Department of Mechanical Engineering, Faculty of Engineering, Istanbul University-Cerrahpasa, Turkey; ^2^Department of Robotics and Intelligent Systems, Institute of Graduate Studies in Science and Engineering, Turkish-German University, Turkey

## Abstract

Finite element (FE) models have frequently been used to analyze spine biomechanics. Material parameters assigned to FE spine models are generally uncertain, and their effect on the characterization of the spinal components is not clear. In this study, we aimed to analyze the effect of model parameters on the range of motion, stress, and strain responses of a FE cervical spine model. To do so, we created a computed tomography-based FE model that consisted of C2-C3 vertebrae, intervertebral disc, facet joints, and ligaments. A total of 32 FE analyses were carried out for two different elastic modulus equations and four different bone layer numbers under four different loading conditions. We evaluated the effects of elastic modulus equations and layer number on the biomechanical behavior of the FE spine model by taking the range of angular motion, stress, and strain responses into account. We found that the angular motions of the one- and two-layer models had a greater variation than those in the models with four and eight layers. The angular motions obtained for the four- and eight-layer models were almost the same, indicating that the use of a four-layer model would be sufficient to achieve a stress value converging to a certain level as the number of layers increases. We also observed that the equation proposed by Gupta and Dan (2004) agreed well with the experimental angular motion data. The outcomes of this study are expected to contribute to the determination of the model parameters used in FE spine models.

## 1. Introduction

Due to the ethical concerns and the requirement of invasive methods, determining the in vivo stress and strain values that occur on the vertebrae under different loading conditions is challenging [1]. The finite element-based computational modeling and simulation approach provide a practical and efficient solution to this problem. By using finite element (FE) analysis, it is possible to simulate the biomechanical behavior of the spinal components and calculate various biomechanical parameters such as stress, strain, and angular motion noninvasively [2–4]. Most of the FE models of the spine are based on computed tomography (CT) data [5]. In the literature, the relationships between the Hounsfield Unit (HU), which is a dimensionless unit used in CT, density, and modulus of elasticity of the anatomical structures were defined through various empirical equations [6–9]. In many FE-based studies, the values of the elastic modulus were calculated by using these equations [10–12], while very few of them focused on the spinal region [9, 13, 14]. The reliability of these equations is still controversial, and a consensus on the use of these equations has not yet been reached [15].

The article "Effect of Model Parameters on the Biomechanical Behavior of the Finite Element Cervical Spine Model" was retracted in 2023. Reasons: signs of a paper mill; compromised peer review; unreliable results or conclusions.

In the literature, the effect of assigned material properties of the ligament, intervertebral disc, and bone tissue on FE analysis results was investigated, but the effect of the number of layers of bone tissues with different material parameters based on HU level was not investigated [16–18]. Kumaresan et al. [17] analyzed the sensitivity of the output of the FE analysis of cervical spinal components including the intervertebral disc, posterior elements, endplates, ligaments, and cortical and cancellous bones to variations in the assigned material properties. They considered the angular motion, intervertebral disc stress, endplate stress, and vertebrae stress as the output of the analysis. They concluded that the effect of changes in material properties of the soft tissues was more determinant than that in the material properties of the bone [17]. However, bone tissue is the main load-bearing structure in the human body, and the mechanical composition of bone tissue should be accurately modeled in a FE analysis to obtain reliable stress and strain levels [19]. In the literature, models were typically separated into three or four layers that are representing vertebral body structures such as the endplates and cortical and cancellous bones [17, 20]. In these studies, the distinction between these tissues was not made considering the level of HU. Rayudu et al. [21] predicted the elastic modulus by taking into account the level of HU, and a vertebra model was built up with nine layers. There is still little knowledge about the required number of layers to be defined for a FE vertebrae model to reflect the actual biomechanical behavior of the bone tissue. Moreover, the question of how sensitive the stress and strain results obtained from FE analyses are to variations in layer numbers and assigned material parameters of the vertebrae has not been answered yet.

In this study, we aimed to analyze the effect of model parameters on the range of motion, stress, and strain responses of a FE cervical spine model. More specifically, we focused on (i) how many layers would be required to obtain an accurate model and (ii) which of the two widely used HU-elastic modulus relationships in the literature would provide a more accurate result in terms of joint range of motion. The FE spinal unit included C2 and C3 vertebrae, intervertebral discs, ligaments, and facets at the same level.

The article "Effect of Model Parameters on the Biomechanical Behavior of the Finite Element Cervical Spine Model" was retracted in 2023. Reasons: signs of a paper mill; compromised peer review; unreliable results or conclusions.

## 2. Materials and Methods

### 2.1. Modeling of the Spinal Unit

CT data of a 55-year-old male cadaver was processed to create the vertebrae model. CT images of the nonpathological cervical spine were obtained from the archive of the Istanbul University-Cerrahpasa, Turkey. The pixel size and slice thickness of the tomography data were 0.49 mm and 0.63 mm, respectively. The spinal functional unit was modeled between the C2 and C3 vertebrae, including the intervertebral disc, ligaments, and facets at the same level. Four different FE vertebrae models were created separately, which were formed from one, two, four, and eight layers depending on HU values (Table 1) [22]. The vertebrae model comprising one layer was defined as a homogenized bone. In the two-layer model, one bone layer was defined for each of the cancellous and cortical bones. In the four-layer model, two bone layers were defined for each of the cancellous and cortical bones. In the eight-layer model, the first three layers were represented as the cancellous bone and the remaining layers were represented as the cortical bone [23]. Bonemat software (Bonemat, BO, Italy) was used to build up the models depending on CT data.

All vertebrae models were assumed to have linearly elastic and isotropic behavior, and their mechanical properties were described by elastic modulus and Poisson's ratio [24]. The material properties for each layer were calculated by taking HU and related density values into account. To do so, the two most common empirical equations for relating HU-elastic modulus in the literature were used to obtain the elastic modulus of the modeled bone tissues [25, 26]. In both studies, CT data were taken from bone samples and compressive force was applied to them. The stress-strain curves were plotted to calculate the elastic modulus. In addition, tissue density measurements were measured. The empirical equations were established between HU, density, and elastic modulus.

Equation (1) was used for the relationships between HU and density (*ρ*) expressed in kg/m^3^ [25, 26]:

(1) $$\begin{array}{c} \rho =0.44\times \text{HU}+527. \end{array}$$

Gupta and Dan [25] proposed the following equation set (equation (2)) to establish the relationships between density (*ρ*) (kg/m^3^) and elastic modulus (*E*) (MPa):

(2) $$\begin{array}{c} E=3\times 10^{-6}\times \rho^{3}\;\text{for }350<\rho \leq 1800,\\ E=1049.25\times 10^{-6}\times \rho^{2}\;\text{for }\rho \leq 350. \end{array}$$

Morgan et al. [26] reported the following equation for the relationship between *ρ* (kg/m^3^) and *E* (MPa):

(3) $$\begin{array}{c} E=4730\times {\left(\frac{\rho }{1000}\right)}^{1.56}. \end{array}$$

Average HU values for all bone layers were specified from CT image data, and the related elastic modulus values were calculated from the abovementioned equations. Poisson's ratio was 0.3 for all models.

The article "Effect of Model Parameters on the Biomechanical Behavior of the Finite Element Cervical Spine Model" was retracted in 2023. Reasons: signs of a paper mill; compromised peer review; unreliable results or conclusions.

The intervertebral disc was modeled to fill the space between the endplates of the vertebrae. The intervertebral disc located between the C2 and C3 vertebrae consisted of the annulus fibrosus and nucleus pulposus layers. The Mooney-Rivlin hyperelastic elements were used to model the annulus ground substance [27]. For the nucleus pulposus, the elastic modulus and Poisson's ratio were 1 MPa and 0.49, respectively, which were reported by Ruberte et al. [27] based on the experimental data available in the literature [28–30].

Anterior longitudinal, posterior longitudinal, facet capsular, supraspinous, interspinous ligaments, and ligamentum flavum were represented by tension-only spring-like connectors with nonlinear material properties (Table 2). The material property of the ligaments was defined in terms of stiffness. The experimentally obtained nonlinear stiffness property was drawn from the literature [31]. Yoganandan et al. [31] measured the tensile force-displacement of all ligaments at different levels of the cervical region.

### 2.2. The Meshing of the Model

The hybrid quadratic tetrahedral element was chosen for the vertebrae and intervertebral disc. The criteria for creating elements influence the number of elements [32]. The geometric criteria of the hybrid quadratic tetrahedral element have been determined such that the lowest volume was 0.3 mm^3^, the lowest internal angle was 10°, and the highest internal angle was 130° [33]. Sizing iterations were carried out up to the longest and shortest side length ratio of 5 and the largest and lowest volume ratio of 2 [33]. All models had 120000 elements (Figure 1).

### 2.3. Loading and Boundary Conditions

Flexion, extension, lateral bending, and axial rotation moments, all of which were 1.5 Nm, were applied to the models [34]. The moment value of 1.5 Nm was assumed to be sufficient to produce motion, but small enough to not injure the tissues [34]. The upper surface of the C2 vertebra was connected to the reference point, which was created in line with the adjacent vertebral body. The moment applied to the reference point was thus distributed over the upper surface of the C2 vertebra. The C3 inferior surface was fixed in all directions. The contact between the intervertebral disc and the endplate was determined to be bounded (slip and clearance were not allowed). The facet joints were coupled between the C2 and C3 vertebrae as a continuum distributing type. For all cases, the loading conditions and analysis were assumed static.

The article "Effect of Model Parameters on the Biomechanical Behavior of the Finite Element Cervical Spine Model" was retracted in 2023. Reasons: signs of a paper mill; compromised peer review; unreliable results or conclusions.

The effects of layer number and elastic modulus on the angular motion, stress, and strain values obtained from the FE analysis of the vertebrae models were compared for four different loading conditions. As a result, a total of 32 analyses (two different elastic modulus equations × four different layer numbers × four different loading conditions) were performed. All analyses were performed by using Ansys software (Ansys, Inc., Canonsburg, PA, USA).

## 3. Results

Angular motion results at the C2/C3 segment were given for four different layer numbers (one, two, four, and eight), two different equations, and four different loading conditions in Figure 2. The model-predicted angular motions were also compared with those obtained from the literature [35]. White and Panjabi [35] analyzed various experimental results from the literature to describe the range of angular motion of the C2-C3 vertebrae. The degree of motion of the C2-C3 vertebrae was experimentally obtained during the same loading conditions that we applied to the models [35]. It can be deduced from Figure 2 that the model-predicted angular motions under flexion, extension, and axial rotation moments were consistent with the experimental data [35]. However, the results obtained for the lateral bending moment were not in agreement with the experimental data. Angular motions obtained by using the equations by Gupta and Dan [25] and Morgan et al. [26] were found similar to each other, especially under the lateral bending moment. The number of layers was found as an effective parameter in the calculation of the angular motion, while the major differences in terms of angular motion were found between one- and two-layer models.

Maximum von Mises stress and strain values that occurred on the C2/C3 intervertebral disc were given in Figure 3. To determine whether the stress and strain values converge to a certain value as the number of layers increases, the stress and strain values obtained from one-, two-, and four-layer models were normalized to those obtained from eight-layer models (Figures 3(a) and 3(b)). When the equation proposed by Gupta and Dan [25] was taken into account, it was seen that the variations in the number of layers led to a 10% change in the stress and 30% in the strain values. As for the equation proposed by Morgan et al. [26], the variations in the number of layers caused a 62% change in the stress and 30% in the strain values. It was also observed that the stress and strain results obtained from four-layer models converged to those of the eight-layer models for both equations.

The article "Effect of Model Parameters on the Biomechanical Behavior of the Finite Element Cervical Spine Model" was retracted in 2023. Reasons: signs of a paper mill; compromised peer review; unreliable results or conclusions.

Table 3 and Table 4 indicate the maximum von Mises stress and strain values that occurred on the vertebrae, respectively. The results were given for each layer and all loading conditions. In Table 3 and Table 4, as the number of layers increases in the first row, the level of HU value for the corresponding layer increases. The first and second values in each cell were based on equation (1) [25] and equation (2) [26], respectively. It was observed from Table 3 that as the layer number in the vertebrae increased, the stress values also increased. In terms of strain values, an opposite trend was observed such that the strain values decreased as the HU value of the layer increased (Table 4). The difference in stress and strain values between layers decreased as the number of layers increased, indicating that more homogenous stress and strain distributions occurred over the vertebrae as the number of layers increased. The use of equation (2) and equation (3) did not result in significant differences between the maximum stress values.

## 4. Discussion

To deepen our understanding of the effect of various surgical interventions on the spinal components, in silico analysis of the spine provides a practical and efficient complimentary solution. Finite element-based in silico analysis has become widespread in the assessment of the spine over the last two decades [15]. The accuracy of such an analysis is critical to obtain clinically meaningful outcomes. In particular, model parameters play an important role in obtaining reliable biomechanical results from spinal FE modeling and simulation studies. The material properties of each element can be assigned depending on the HU value. On the other hand, such a methodology would lead to a high computational cost and errors due to discontinuities in the internal structures of the bone tissue. Therefore, there are many studies in the literature defining the vertebral bone into different layers, namely cortical and trabecular bone layers [36, 37]. Accordingly, we aimed to analyze the effects of variations in elastic modulus and layer number on the model-predicted angular motion, stress, and strain values that occurred at the C2/C3 level of the FE spine model under various loading modes. We also compared the model-predicted angular motion with the experimentally obtained data. The strain and stress values on the intervertebral disc and vertebrae were separately evaluated.

Angular motions under flexion and extension moments occurred in a similar range (Figure 2), and they agreed with the experimental data [35], indicating that the mechanical properties of the disc structure were well defined. The model-predicted angular motion under the lateral bending moment was lower than the experimental data, which indicates that the stiffness value assigned to the FE model in the direction of the lateral bending movement was quite high. The facet joint influences the lateral bending motion considerably [38], and hence the low level of model-predicted motion may be attributed to the uncertainty of the assigned mechanical properties of the facet joint. Under the axial rotation moment, the calculated angular motion from the FE analysis was within the range of the experimentally obtained data. In the literature, it was reported that the level of angular motion is highly associated with the material properties of the soft tissues [39]. The results of our study showed that the soft tissues except facets were well defined in the FE model.

The article "Effect of Model Parameters on the Biomechanical Behavior of the Finite Element Cervical Spine Model" was retracted in 2023. Reasons: signs of a paper mill; compromised peer review; unreliable results or conclusions.

Angular motions of the one- and two-layer models had a greater variation than those in the models with four and eight layers (Figure 2). This result indicates that defining the vertebrae with the cancellous bone caused a big effect on the angular motion results. Unlike the one-layer model, the two-layer model characterized the cancellous bone. It was observed that the angular motion level converged to a certain degree as the number of layers increased. The angular motions obtained for the four- and eight-layer models were almost the same, indicating that the use of a four-layer model would be sufficient to achieve the stress value converging to a certain level as the number of layers increases.

Figure 3 illustrates how many numbers of layers would be adequate to define the vertebrae. It was revealed that the change in the material properties of the vertebrae plays a decisive role in the stress and strain values over the intervertebral disc. When the stress and strain on the intervertebral disc structure are examined in Figures 3(a) and 3(b), it was observed that the results of the model using both equations with four layers converged to the results of the model with eight layers.

The difference in stress and strain distributions between the layers decreased as the number of layers increased (Table 3 and Table 4). The stress and strain results obtained by using equation (2) and equation (3) on the one-layer vertebrae model were quite similar. However, the variation in the results was greater between equation (2) and equation (3) when the number of layers increased. When compared to the cortical bone, the experimental mechanical testing on the vertebrae specimens showed that the strain level in the cancellous bone was higher and the stress level in the cancellous bone was lower [40, 41]. It was observed from the stress results of our study that equation (2) agreed more with the experimental data than equation (3). The fact that Gupta and Dan [25] created separate sets of equations for the cancellous and cortical bone may have led to results that are more consistent with experimental data. When the stress values of the vertebra are examined, it was observed that the stress levels in some layers decreased as the elastic modulus of the layer increased, which is not compatible with the literature [41].

The article "Effect of Model Parameters on the Biomechanical Behavior of the Finite Element Cervical Spine Model" was retracted in 2023. Reasons: signs of a paper mill; compromised peer review; unreliable results or conclusions.

In 2001, Morgan and Keaveny reported in their experimental study on cadavers that the yield stress of the cancellous bone during compression was 2.02 MPa, the yield strain was 0.77%, the yield stress was 1.72 MPa, and the yield strain during tensile was 0.70% [40]. In addition, the cortical bone with a modulus of elasticity of 18 GPa had a yield stress of 70 MPa and a yield strain of 0.55% [41]. When these experimental values are taken into account, it was seen that the stress and strain values obtained from the models with one and two layers exceeded the experimentally obtained stress and strain values over the cancellous bone. On the other hand, the eight-layer model provided more comparable results to the experimental data. When the model-predicted stress results from the cortical bone were considered, it was seen that all stress values remained within the specified range defined by the experiments [41]. In terms of strain value, it was observed that the models with four and eight layers provided more accurate results.

Studies on the investigation of the density and elastic modulus relationship for different bone structures are very few [25, 26]. The relationship between elastic modulus and apparent density does depend on the anatomic site, which was also experimentally proven by Morgan et al. [26]. Also, the empirical relations used for defining elastic modulus are not only anatomical site specific, they can also vary between patients and computed tomography (CT) scan machine. Although these limitations are present in creating the finite element bone models, these models are most often derived from CT data in the literature [42]. Equation (2) was empirically obtained based on the CT data of the scapula [25]. On the other hand, Morgan et al. [26] carried out their experimental study on different bone structures including vertebrae. The limitation in [26] is that the authors did not provide separate equations for the cancellous and cortical bones depending on the individual bone density, but rather a single equation was developed to reflect the mechanical properties of the entire bone structure.

The article "Effect of Model Parameters on the Biomechanical Behavior of the Finite Element Cervical Spine Model" was retracted in 2023. Reasons: signs of a paper mill; compromised peer review; unreliable results or conclusions.

There are some limitations to our study. First, we only focused on the C2/C3 segment of the spine in our study since well-defined and comparable experimental data were available for this segment. However, the anatomical and functional differences available in the vertebrae can influence the obtained results. Moreover, the spine model used in our study would not represent various pathological bone conditions such as osteoporotic bone. Therefore, more FE models characterizing different bone conditions are needed to be investigated. Second, to reduce the calculation burden and provide condensed and experimentally compared results, we did not perform dynamic analysis. However, the assigned mechanical properties of the vertebrae would play a critical role under the dynamic loading of the tissue. Third, due to the lack of well-defined experimental data, all vertebrae models were assumed to have linearly elastic and isotropic behavior, which would not perfectly reflect the mechanical characteristics of the tissues. Fourth, the cadaver samples from which the experimental data were obtained and the CT data from which the FE models were created were different. However, the experimental and modeling/simulation works should be ideally carried out on the same cadaveric specimen, but that was not possible in our study due to technical limitations in terms of obtaining a fresh cadaver. And, lastly, since -FE analyses were implemented to only one sample of the vertebral body, caution should be taken when interpreting and generalizing the results obtained from our study.

## 5. Conclusion

We aimed to analyze the effect of model parameters on the range of motion, stress, and strain responses of the FE cervical spine model. We concluded that the angular motions of the one- and two-layer models had a greater variation than those in the models with four and eight layers. The angular motions obtained for the four- and eight-layer models were almost the same, indicating that the use of a four-layer model would be sufficient to achieve the stress value converging to a certain level as the number of layers increases. We also observed that the equation proposed by Gupta and Dan in 2004 agreed well with the experimental data because the cortical and cancellous bones were modeled separately. In the next step, we plan to investigate the effects of assigned mechanical parameters on the response of the entire spine model under dynamic loading conditions.

## Figures and Tables

**Figure 1:** Finite element model of the C2 and C3 vertebrae and intervertebral disc.

**Figure 2:** Angular motion at the C2/C3 joint for four different layer numbers (one-, two-, four-, and eight-layer models), two different equations (equation (2) and equation (3)), and four different loading conditions (flexion, extension, lateral bending, and axial rotation moments). The results based on equation (2) were represented by a solid line with a circle [25] and those based on equation (3) by a solid line with a triangle [26]. Experimentally obtained angular motions were represented by grey zones [35].

The article "Effect of Model Parameters on the Biomechanical Behavior of the Finite Element Cervical Spine Model" was retracted in 2023. Reasons: signs of a paper mill; compromised peer review; unreliable results or conclusions.

**Figure 3:** Maximum normalized stress (a) and strain (b) values on the C2/C3 intervertebral disc. The stress and strain values obtained from one-, two-, and four-layer models were normalized to that obtained from eight-layer models. The results based on equation (2) were represented by a solid line with a circle [25] and those based on equation (3) by a solid line with a triangle [26].

**Table 1:** Generated finite element vertebrae models consisted of different layer numbers depending on HU values of the cortical and cancellous bone.

Range of HU values defined for the corresponding finite element vertebrae models			
One-layer model	Two-layer model	Four-layer model	Eight-layer model
148-1988	148-661 662-1988	148-300 301-661 662-1300 1301-1988	148-300 301-500 501-661 662-900 901-1100 1101-1300 1301-1600 1601-1988

**Table 2:** The force of ligaments relative to the displacement [31].

Anterior longitudinal		Posterior longitudinal		Facet capsular		Interspinous ligaments/supraspinous		Ligamentum flavum	
Force (N)	Displacement (mm)	Force (N)	Displacement (mm)	Force (N)	Displacement (mm)	Force (N)	Displacement (mm)	Force (N)	Displacement (mm)
32.5	1.24	26.8	1.02	59.5	2.02	8.6	1.38	29.2	1.71
60.8	2.46	49.5	2.12	122.8	4.00	16.9	2.74	54.9	3.37
82.4	3.63	65.0	3.13	170.2	5.92	22.7	4.12	71.9	5.10
100.3	4.78	79.8	4.23	206.5	7.99	28.8	5.55	94.5	6.68

**Table 3:** The maximum von Mises stress values on the vertebrae. The first and second values in each cell are based on equation (1) [25] and equation (2) [26], respectively.

Maximum von Mises stress value (MPa)									
Number of layer		1	2	3	4	5	6	7	8
Flexion	One-layer model	17.8/19.0							
	Two-layer model	12.1/20.0	27.2/25.0						
	Four-layer model	4.9/7.0	15.5/23.8	19.4/20.2	26.7/26.0				
	Eight-layer model	5.8/9.0	7.0/9.7	7.9/14.1	13.3/25.8	16.3/18.6	24.0/23.6	23.7/23.9	17.8/18.7

Extension	One-layer model	17.8/20.0							
	Two-layer model	12.1/21.0	26.7/25.4						
	Four-layer model	4.9/7.0	16.5/24.8	20.4/20.9	33.4/26.9				
	Eight-layer model	5.8/7.1	7.0/9.7	8.5/14.7	14.1/26.9	17.1/19.7	25.5/24.5	28.9/24.8	17.7/19.8

Lateral bending	One-layer model	13.5/13.8							
	Two-layer model	10.3/5.8	24.4/0.4						
	Four-layer model	4.4/7.4	13.5/15.0	15.4/12.1	24.7/23.1				
	Eight-layer model	2.1/1.9	5.3/8.1	11.3/13.4	18.3/18.1	14.2/12.0	16.3/12.9	27.5/18.9	18.8/23.1

Axial rotation	One-layer model	9.3/9.3							
	Two-layer model	5.4/10.1	12.4/11.1						
	Four-layer model	3.7/5.7	7.6/8.3	9.5/9.0	14.2/10.2				
	Eight-layer model	2.4/2.5	4.2/6.4	5.6/7.3	8.1/9.9	9.6/11.3	10.3/13.6	12.2/14.2	12.7/10.7

The article "Effect of Model Parameters on the Biomechanical Behavior of the Finite Element Cervical Spine Model" was retracted in 2023. Reasons: signs of a paper mill; compromised peer review; unreliable results or conclusions.

**Table 4:** The maximum strain (%) values on the vertebrae. The first and second values in each cell are based on equation (1) [25] and equation (2) [26], respectively.

Maximum strain value (%)									
Number of layer		1	2	3	4	5	6	7	8
Flexion	One-layer model	1.1/1.2							
	Two-layer model	1.9/1.1	1.0/0.8						
	Four-layer model	1.1/0.4	1.6/0.9	1.0/0.6	0.3/0.5				
	Eight-layer model	0.8/0.3	1.0/0.4	0.7/0.7	0.6/0.7	0.6/0.6	0.4/0.6	0.4/0.5	0.2/0.2

Extension	One-layer model	0.8/1.0							
	Two-layer model	1.2/0.7	0.7/0.6						
	Four-layer model	1.6/0.6	1.0/0.6	0.6/0.5	0.4/0.5				
	Eight-layer model	1.1/0.7	0.6/0.4	0.9/0.6	0.9 0.6	0.7/0.6	0.6/0.5	0.4/0.5	0.4/0.2

Lateral bending	One-layer model	0.8/0.8							
	Two-layer model	1.5/0.6	0.8/0.4						
	Four-layer model	1.0/0.4	1.2/0.4	0.7/0.3	0.4/0.2				
	Eight-layer model	0.4/0.1	0.9/0.4	1.2/0.5	1.4/0.6	0.8/0.3	0.4/0.2	0.3/0.2	0.3/0.2

Axial rotation	One-layer model	0.5/0.5							
	Two-layer model	0.7/0.3	0.3/0.2						
	Four-layer model	0.7/0.3	0.6/0.3	0.3/0.2	0.3/0.2				
	Eight-layer model	0.5/0.2	0.6/0.3	0.6/0.2	0.5/0.3	0.4/0.2	0.3/0.2	0.3/0.1	0.2/0.1

## Data Availability

No data is available.
